# Oxidized Low-density Lipoprotein (ox-LDL) Cholesterol Induces the Expression of miRNA-223 and L-type Calcium Channel Protein in Atrial Fibrillation

**DOI:** 10.1038/srep30368

**Published:** 2016-08-04

**Authors:** Fengping He, Xin Xu, Shuguo Yuan, Liangqiu Tan, Lingjun Gao, Shaochun Ma, Shebin Zhang, Zhanzhong Ma, Wei Jiang, Fenglian Liu, Baofeng Chen, Beibei Zhang, Jungang Pang, Xiuyan Huang, Jiaqiang Weng

**Affiliations:** 1 Department Institute of Cardiovascular Diseases, The Yuebei People’s Hospital, Medical College, Shantou University, Shantou, Guangdong, China

## Abstract

Atrial fibrillation (AF) is the most common sustained arrhythmia causing high morbidity and mortality. While changing of the cellular calcium homeostasis plays a critical role in AF, the L-type calcium channel α1c protein has suggested as an important regulator of reentrant spiral dynamics and is a major component of AF-related electrical remodeling. Our computational modeling predicted that miRNA-223 may regulate the *CACNA1C* gene which encodes the cardiac L-type calcium channel α1c subunit. We found that oxidized low-density lipoprotein (ox-LDL) cholesterol significantly up-regulates both the expression of miRNA-223 and L-type calcium channel protein. In contrast, knockdown of miRNA-223 reduced L-type calcium channel protein expression, while genetic knockdown of endogenous miRNA-223 dampened AF vulnerability. Transfection of miRNA-223 by adenovirus-mediated expression enhanced L-type calcium currents and promoted AF in mice while co-injection of a *CACNA1C*-specific miR-mimic counteracted the effect. Taken together, ox-LDL, as a known factor in AF-associated remodeling, positively regulates miRNA-223 transcription and L-type calcium channel protein expression. Our results implicate a new molecular mechanism for AF in which miRNA-223 can be used as an biomarker of AF rheumatic heart disease.

Atrial fibrillation (AF) is induced by wide range of factors^1^,^2^ including atrial dilation, oxidative stress, atrial ischemia or hypoxia, calcium (Ca^2+^)-handling abnormalities, and intracellular Ca^2+^ overload. It can cause or exacerbate heart failure and is also a high risk factor of ischemic stroke from thromboembolism^3^. AF can be characterized by the alteration of electrophysiology as a result of so called “atrial remodeling” which promotes persistent AF even in the absence of progressive underlying heart disease^4^,^5^. This remodeling process has been suggested to be associated with the expression of L-type Ca^2+^ channels^6^. Numbers of studies have shown that oxidative stress contributes to the pathogenicity of cardiovascular diseases^7^. Indeed, ox-LDL or lysophosphatidylcholine (LPC) increases oxidative stress by generating reactive oxygen species (ROS) which cause changes in the electrophysiological properties of cells^8^. Ox-LDL have been shown to mediate the increase of the L-type Ca^2+^ current (I_CaL_) as well as the sarcoplasmic reticulum (SR) Ca^2+^-load in which they may relate to the upregulation of the intracellular Ca^2+^ concentrations ([Ca^2+^]_i_), the occurance of early afterdepolarizations (EADs) and delayed afterdepolarizations (DADs) in human AF^9^. Alterations of transmembrane sodium (Na^2+^) and potassium (K^+^) fluxes also contribute to the changes in electrophysiological properties in response to the ox-LDL^10^. Interestingly, elevation of ox-LDL in plasma has shown to associate with atherosclerosis by mediating atherogenic processes in vascular myocytes^11^. In addition, ox-LDL enhances I_Ca, L_ via LPC-induced mitochondrial ROS production in cardiac myocytes, which in turn mediates a response in native Ca^2+^ currents (I_Ca_)^12^.

Recent studies have demonstrated that miRNAs play an important role for regulating cardiac excitability and arrhythmogenesis in various cardiac diseases, including myocardial infarction^13^, cardiac hypertrophy^14^, diabetic cardiomyopathy^15^, AF^16^ and other cardiac conditions^17^. Studies have primarily focused on the muscle-specific miRNAs such as miRNA-1 and miRNA-133, with the exception of miRNA-26, and miRNA-328, which contribute to shapen the cardiac electrophysiology^18^,^19^,^20^. In particular, changing of miR-223 expression has recently been reported in rheumatic heart disease and other diseases^16^,^19^. Up-regulation of miRNA-223 alters prostate cancer pathways (such as trial ischemia or hypoxia, Ca^2+^-handling abnormalities, intracellular Ca^2+^ overload, and expression of L-type Ca^2+^ channel proteins) by targeting the “seed” regions that bind to the complementary sequences of the 3′ untranslated regions (UTR)^21^,^22^. However, the involvement of miRNA-223 in the cardiovascular diseases is not yet well understood. In this study, we aim to investigate the role of ox-LDL on the regulation of miRNA-223 and L-type Ca^2+^ channel protein during atrial fibrillation.

## Results

### Expression profile of miRNAs during AF in the canine model

We first aimed to understand the expression of miRNAs during AF by using a well-established canine model with induced atrial fibrillation by A-TP. A-TP increased the vulnerability to AF as shown by facilitated AF induction by electrical stimuli, and prolonged duration of electrically induced AF (Fig. 1A). The cellular and ionic alterations were also consistent to the atrial remodeling during AF (Fig. 1). Using this canine AF model, we detected miRNAs in atrial tissue by quantitative real-time reverse-transcription polymerase chain reaction (qRT-PCR), and compared the expression of the miRNAs between the dogs from control and AF groups. Three miRNAs (miRNA-21, miRNA-133, and miRNA-223) were identified by qRT-PCR showing significant upregulation of miRNA-223 by more than 50%. No significant change was observed from the levels of miRNA-21 and miRNA-133 (Fig. 1E,F).

### Clinical characterization of the patients with NSR and AF

Of the 200 patients in our study, 110 (55%) were female, with a median age of 45 years (ranging from 21–75 years). 93 (46.5%) were diagnosed with NSR (chronic rheumatic MS without AF) and 107 (53.5%) with AF (chronic rheumatic MS with AF). There is a significant difference in age between the NSR and AF groups (*P* < 0.05). Preoperative color Doppler echocardiography showed that the left atrial size of the patients with AF is significantly greater compared to those with NSR (*P* < 0.01).

### Ox-LDL induces the Ca^2+^ channel protein and miRNA-223 expression

In cultured H9c2 cells, ox-LDL treatment produced an activated phenotype of elongated myocardial cells (Fig. 2A). Moreover, ox-LDL increased miRNA-223 expression by approximately 4-fold (Fig. 2B,C). To further understand the relationship between the miRNA-223 and ox-LDL, we determined the role of miR-223 expression in H9c2 cells upon ox-LDL treatment. MiRNA-223 was first transfected into H9c2 cells. The cells were then stimulated by 25 and 50 μg/mL ox-LDL for 10, 20, 40, or 60 min (Fig. 2B,C). MiRNA-223 overexpression upregulated [Ca^2+^]_i_ and further promoted ox-LDL-induced upregulation of [Ca^2+^]_i_ in a dose-and time-dependent manner (Fig. 2D). Cav1.2 protein was significantly increased by 30 min of ox-LDL (25 μg/mL) treatment (Fig. 2E). Western blot analysis showed markedly increase of Cav1.2 protein levels in the myocardial cells of the Tg mice with miRNA-223 overexpression. Higher level of Cav1.2 was detected in Tg mice upon exposure to ox-LDL than the mice in control (NC) and AMO-223 groups (Fig. 2F). Our model predicted simultaneous depolarization-induced I_Ca, L_ and Ca^2+^ transients in fluo-3- loaded myocytes. Atrial myocytes were preconditioned for 1 min using the I_Ca,L_ activation protocol in all subsequent voltage-clamp experiments. As a result of SR Ca^2+^ release, ox-LDL (25 μg/mL for 30 min) caused a rapid increase in [Ca^2+^]_i_ (Fig. 1 in the online-only Data Supplement).

### The involvement of miRNA-223 during AF

We then determined that if the AF is regulated by miRNA-223. To test this hypothesis, two miRNA-223 loss-of-function approaches were adopted. In the first approach, we generated Tg mouse line (AMO/Tg) expressing miRNA-223 antisense to genetically knockdown the endogenous miRNA-223. In the second approach, we injected anti-miRNA-223 into wild type mice to knockdown the endogenous miRNA-223. The mice were first pretreated with low-dose carbachol through the tail vein for seven consecutive days before inducing AF by intracardiac pacing (Fig. 3). AF induction was substantially dampened in adenovirus (adv)-miRNA- 223-treated WT mice (Fig. 3A). The reduced number of animals with successful AF induction by electrical stimulation and sham-operated, age-matched mice are also shown (Fig. 3B). Adenovirus vector without miRNA-223 (adv-miR-free) knockdown in WT mice was used as the NC (Fig. 3C). Similar changes were not observed in WT mice or mismatched AMO/Tg mice (Fig. 3D). Quantitative RT-PCR confirmed that miRNA-223 levels were two times higher in the AF group than the non-AF group. Levels of miRNA-21 and miRNA-133 remained no change in the AF group (Fig. 3E) while the miRNA-223 level reciprocally decreased by 2-fold in the miRNA-223 knockdown mice (Fig. 3F).

### *CACNA1C* gene as the miR-223 target

We next delineated the target gene of miR-223 which plays a key role in AF and the associated electrical remodeling process. Our computational analysis suggested that miR-223 regulates the *CACNA1C* gene as it contains multiple sequence motifs complementary to the “seed site” of miR-223 in its 3′ UTR and coding regions (Fig. 2 in the online-only Data Supplement). To determine *CACNA1C* as the cognate target of miR-223, we cloned the fragments containing *CACNA1C*-miR-223 binding sites into the 3′ UTR of the luciferase gene for luciferase reporter activity assay. Transfection of miR-223 (10 nmol/L) with constructs carrying different target fragments caused enhancement of luciferase activity (Fig. 4A). The reduction was efficiently rescued in the presence of AMO-223 (10 nmol/L). The induction of *CACNA1C* by mi-223 was further verified by western blotting in neonatal mouse atrial myocytes transfected with miR-223 (Fig. 4B). In addition, Cav1.2 protein level was significantly increased in atrial tissues from A-TP dogs (Fig. 4C). The level of control protein, connexin 43 remained no change between different groups of condition. Upregulation of Cav1.2 protein levels was also observed in miR-223/Tg rats (Fig. 4D). Similar effect of miR-223 on *CACNA1C* transcription was also found in miR-223/Tg mice and cultured neonatal rat atrial myocytes. MiR-223 induced higher than 50% in *CACNA1C* transcript levels and significant upregulation of Cav1.2 protein levels was observed in AF patients (Fig. 4E). Ox-LDL regulates miR-223 expression by directly targeting its 3′ UTR. 3′ UTR of miR-223 mRNA contains two highly conserved binding sites (from positions 35–57 and 1743–1765) (Supplement Figure 2). Computational modeling has shown that both sites increased SR Ca^2+^-load and RyR2 dysregulation contributes to spontaneous diastolic SR Ca^2+^-release events in cardiomyocytes from AF patients and A-TP dogs^23^,^24^. Similar to vasoactive agonists (e.g., ATP, histamine and bradykinin) that increase [Ca^2+^]_i,_ and I_Ca,L_ in myocyte cells^25^. Our results suggest that upregulation of miRNA-223 by ox-LDL is activated by the increase of [Ca^2+^]_i_ in myocyte cells.

We also observed that miR-223 decreased myocardial constriction and induced myocardial cell apoptosis. The level of miR-223 was previously shown to be increased in animals and humans with AF exposed to ox-LDL, which promoted myocardial cell apoptosis^26^. It is possible that these actions result from the regulation of distinct apoptotic and constriction factors by miR-223 repress IGF-1R. Based on computational analysis, we also identified putative binding sites in the 3′-untranslated regions (3′ UTR) of IGF-1R, which might bind the miR-223 seed sequence (Supplement Figure 4).

## Discussion

In this study, we showed that miRNA-223 and Cav1.2 protein expression are upregulated during AF conditions (Figs 1 and 2). Ox-LDL induced the transcription of miRNA-223 (Figure S2) and thereby promoted the Cav1.2 expression by activating ROS and regulating the Ca^2+^-release. This mechanism may occur in atrial myocytes, which show pronounced electrophysiological and pathophysiology remodeling during AF^23^,^24^,^25^,^27^,^28^. Ox-LDL has been reported to alter calcium handling in vascular and cardiac myocytes^29^,^30^, which may explain why it induces a broad spectrum of effects ranging from mild to severe AP prolongation, the occurrence of EADs, DADs and the abnormal spontaneous activity to cell death in the same incubation fraction^30^. Our computational prediction and experimental results indicate that miRNA-223 regulates L-type Ca^2+^ channel under specific disease conditions.

Here, we performed simultaneous recordings of Ca^2+^ and membrane currents (or potentials) induced by ox-LDL in atrial myocytes. We observed >3 and >1.5-folds increase of Cav1.2 and Cavβ1 protein, respectively, the two hallmarks of atrial remodeling. In addition, miRNA-223 triggered >3-fold I_Ca,L_ amplitudes and a tendency towards higher diastolic [Ca^2+^]_i_ in AF patients than controls. Importantly, we found that myocytes from AF patients and the canine AF model show increased miRNA-223 expression, accompanied by greater I_Ca, L_ amplitudes. L-type Ca^2+^ channel protein expression was downregulated in AF patients and the canine AF model (similar to Ca^2+^ channel deregulation reported previously^19^,^20^) highlighting the ability of ox-LDL (or LPC, an ox-LDL component) to differentially regulate Ca^2+^ currents, possibly by different mechanisms depending on the length and concentration of ox-LDL exposure. Our findings also suggest that the activation of Ca^2+^ current by ox-LDL is induced by a [Ca^2+^]_i_-dependent mechanism^27^. Intriguingly, ox-LDL enhanced miRNA-223 expression has frequently been implicated in AF promotion, and suggested to couple rapid atrial activity to atrial remodeling via ROS and Ca^2+^-sensitive signaling via calcineurin^26^,^28^,^31^.

We demonstrated that miRNA-223 targets *CACNA1C* to enhance I_Ca,L_ and shorten the action potential duration in atrial myocytes (Fig. 4). Here, we showed that ox-LDL exposure increases both miR-223 and Cav1.2 expression. Moreover, Ca^2+^ flux in cultured myocytes is accelerated by miR-223. Studies using confocal microscopy has identified a role for miR-223 in L-type calcium channel activity^21^,^32^, because the L-type calcium channel is the principal Ca^2+^ entry pathway in myocytes^33^. Our results from luciferase assay showed that *CACNA1C* is a direct target of miR-223 (Fig. 4A). Taken together, these results suggest that ox-LDL induces the expression of Cav1.2 via miR-223. Another major strength of our study is that our results implicate that miR-223 in the attenuation of AF remodeling relates to Ca^2+^-handling abnormalities. Computational analyses showed that Ca^2+^- dependent concentration and Ca^2+^-handling abnormalities are critical AF-promoting factors^34^. Moreover, miRNA-223 increases the L-type Ca^2+^ channel proteins supports a [Ca^2+^]_i_-dependent mechanism in Ca^2+^ current activation by ox-LDL^35^,^36^. We confirmed the relationship between miRNA-223 and ox-LDL changes in a dose-and time-dependent manner (Fig. 2B,C). Ox-LDL results in almost immediate activation of miR-223, which is the major cellular pathway to ox-LDL production. The ability of antagomiR-223 to rescue miRNA-223-Tg mice from the AF phenotype and associated atrial remodeling properties, suggests miRNA-223’s potential as a target for molecular conversion of AF to a sinus rhythm (Fig. 3). Normalization of miRNA-223 levels may be a novel strategy for converting AF to a sinus rhythm in the clinical setting. In this sense, the antagomiR approach represents a wise choice, as this technique has been reported to have superior cellular stability and miRNA specificity under *in vivo* conditions^37^,^38^. Recently, lectin-like ox-LDL receptor (LOX-1) was shown to be up-regulated in cardiac myocytes during ischemia/reperfusion. Following activation by ox-LDL, LOX-1 was also found to affect the extent of myocardial injury by inducing oxidative stress in cardiac myocytes^39^, which is known to be related to inflammation in AF^40^,^41^,^42^,^43^.

Our results implicate the role of miR-223 in AF pathophysiology and pathogenesis. *In vivo*, electrical remodeling and alterations of Ca^2+^ signaling are likely to act together to induce arrhythmia and AF. Indeed, the probability of APs and APD reaching the AP threshold for any given magnitude of spontaneous Ca^2+^ release which revealed a significant ox-LDL-induced increase in Ca^2+^ currents^44^. Here, we observed electrophysiological alterations including APs, APD, EADs, DADs, and spontaneous activity (Figure S1C), which are known to be potentially trigger arrhythmias. Our results also revealed that the left ventricular ejection fraction of the AF group was significantly decreased compared with the NSR group, where a significant negative correlation was observed between the plasma level of ox-LDL and the left ventricular ejection fraction^45^. This finding suggests that LDL oxidation may take place in the myocardium, which would further imply the existence of a higher ox-LDL concentration in the myocardium compared with the plasma.

We have discovered that miRNA-223 regulates the *CACNA1C* gene and its encoded L-type Ca^2+^ channels. MiRNA-223 is consistently increased in AF patients and animal AF models, and AF-related miRNA-223 upregulation is likely due to enhancement of miRNA-223 transcription by ox-LDL. These findings provide a new insight into the molecular mechanisms underlying the common and important tachyarrhythmic AF, and may have implications for other arrhythmia conditions with dysregulated Ca^2+^ currents^46^,^47^. Thus, miRNA-223 may be used as a novel biomarker for diagnosing AF vulnerability and early phase AF of rheumatic heart disease.

## Materials

The methods were carried out in accordance with the relevant guidelines, included Atrial fibrillation induction in mice model, Establishment of a canine AF model, Collection of atrial samples from patients with AF, Adenovirus construction and infection, Luciferase reporter assay, Quantitative RT-PCR.

### Atrial fibrillation induction in mice model

All animal experiments preformed in the study were approved by the Experimental Animal Administration and Ethics Committee of the Medical College of Shantou University, China. Wild-type (WT) C57BL/6 mice were divided into two groups: control (Ctl) (*n* = 10) group and antagomiR-223 (*n* = 10) group. Intracardiac pacing was performed by inserting an 8-electrode catheter through the jugular vein to the right atrium and ventricle^6^. Inducibility of atrial arrhythmias was tested by applying 6-second bursts through the catheter electrode using an automated stimulator which was a part of the data acquisition system. Next, 50 μg/kg of carbachol was injected through the jugular vein. Two minutes later, the same burst combination was applied to the mice. AF was considered inducible if the burst stimulus produced a period of rapid irregular atrial rhythm and lasted for at least 1 second or more, calculated from direct atrial activation recordings.

### Establishment of a canine AF model

Two mongrel dogs of either gender, weighing around 15 kg were anesthetized by intravenous pentobarbital sodium (30 mg/kg^−1^) and implanted with right atrial pacemakers. Atrial fibrillation was induced by a maximum of 8 weeks atrial tachypacing (A-TP) at 400 bpm. Dogs with spontaneously persisting AF were used for the study. All animal experiments preformed in the study were approved by the Experimental Animal Administration and Ethics Committee of the Medical College of Shantou University, China.

### Collection of atrial samples from patients with AF

Collection of human LAA tissues and the procedures were approved by the Ethics Committee of the Affiliated Yuebei Hospital of Shantou Medical College. Informed consent was obtained from all subjects. The gene and protein expression from the LAA tissue samples were analyzed by qRT-PCR and western blotting respectively (Supplementary Methods).

### Adenovirus construction and infection

The recombinant adenovirus was carried out in accordance with the previous study reported by van Rooij *et al*.^48^. In brief, Rno– miRNA-223 precursor DNA (5′-GGATCCgACCCCGTCCCCCCGTCCTCCC CGAGTCCCTCTTTCGTAGATGTCGG GGACCGGGAGAGACGG GAAGGCAGGGGACAGGGGTTTAttttttAAGCTT-3′) was synthesized (GenScript, Shanghai, China) and inserted into the adenovirus shuttle plasmid pDC316-EGFP-U6 (Microbix Biosystems Inc., Mississauga, ON, Canada). pDC316-EGFP-U6 was then co-transfected with the infectious adenovirus genomic plasmid (pBHGloxΔE1, 3Cre) into H9c2 cells using liposome transfection reagent to generates a recombinant adenovirus (Fig. 3).

### Luciferase reporter assay

The luciferase assay was carried out in accordance with the previous description^21^,^33^. In brief, H9c2 cells were transfected with the pMIR- REPORT luciferase miRNA expression reporter vector carrying the 3′ UTR of *CACNA1C* or pGL3 and the promoter-luciferase fusion plasmid. The cells were cultured in 48-well plates for 48 hours at 37oC with 5% CO2. Dual-LuciferaseH Reporter Assay System (Promega, DLRTM, E1960, USA) was carried out in accordance with the manual instructions. Renilla luciferase intensity was used as internal control to normalize the luminescence intensity of Firefly luciferase^47^,^48^.

### Quantitative RT-PCR

Total RNA was reverse-transcripted using QuantiTect Reverse Transcriptase (Qiagen). qRT-PCR was performed using the CFX96TM real-time (RT) PCR System (BIO-RAD, USA) (Supplementary Methods).

### Data analysis

Statistical analyses were performed using SPSS 19.0 software. Data are expressed as mean ± SEM. Statistical comparisons among multiple groups were performed by analysis of variance (ANOVA). *t*-test with Bonferroni correction was used for the Ca^2+^ channel data. Age-matched comparisons between control and patient groups were performed using unpaired Student *t* tests. Group comparisons for AF incidence were performed using the χ^2^ test. Two-tailed *P* < 0.05 indicated statistically significant differences.

## Additional Information

**How to cite this article**: He, F. *et al*. Oxidized Low-density Lipoprotein (ox-LDL) Cholesterol Induces the Expression of MiRNA-223 and L-type Calcium Channel Protein in Atrial Fibrillation. *Sci. Rep.* **6**, 30368; doi: 10.1038/srep30368 (2016).

## Supplementary Material

Supplementary Information

## Figures and Tables

**Figure 1:** Characterization of the canine AF model. AF was induced by A-TP for 8 weeks. AF was induced by a single premature extrastimuli at a basic pacing cycle length of 300 msec. (**A**) Verification of AF vulnerability. Left, representative direct atrial activation recordings obtained from the left atrial wall of a control (Ctl) dog with sinus rhythm, and an A-TP dog (AF). Right, averaged data of AF incidence and duration. AF incidence was the number of animals demonstrating at least one run of induced AF, and AF duration was measured once induced. *P < 0.05 vs Ctl, unpaired t test; n = 5 dogs in each group. (**B,C**) Verification of atrial electrical remodeling. Note that I_Ca, L_ is significantly upregulated in A-TP dogs. *P < 0.01 vs Ctl. (**D**) Enhancement of I_Ca, L_ density (I_Ca, L_, pA/pF) in A-TP animals relative to Ctl. Action potentials were recorded in single, freshly isolated atrial myocytes using the current-clamp mode in the whole-cell patch-clamp configuration. I_Ca, L_ was recorded using the voltage-clamp mode in the whole-cell patch-clamp configuration; the voltage protocols are shown in the inset. *P < 0.05 vs Ctl, unpaired t test; n = 20 cells in each group. (**E**) qRT-PCR verification of upregulated miRNA-223 expression in A-TP dogs, using miR-1 as a negative control. *P < 0.001 vs. Ctl. The negative controls, miR-21 and miR-133, were unaltered in A-TP dogs. (**F**) qRT-PCR verification of upregulated miRNA-223 expression in AF patients, using miR-1 as a negative control. *P < 0.001 vs. Ctl. The negative controls, miR-21 and miR-133, were unaltered in AF patients.

**Figure 2:** Ox-LDL induces increased of Ca^2+^ channel protein and miRNA-223 expression. (**A**) The control group (left) of myocardial cells was not been treated with ox-LDL and does not show lipid constituent based fluorescence with laser scanning confocal microscopy. The AF group (right) showed that in ox-LDL treated myocardial cells, transfection efficiencies >80% were detected by fluorescence microscopy, which are suggestive of increased ox-LDL production by 50 μg/mL ox-LDL for 60 min. (**B,C**) Enhanced miRNA-223 expression was induced by ox-LDL. A “dose-response” relationship between miRNA-223 and ox-LDL levels was observed. Bars represent mean ± SD of quantitative densitometric analyses from three separate experiments. **P < 0.001 vs. Ctl, *P < 0.01 vs. Ctl, ^†^*P* < 0.05 vs. Ctl. (**D**) Effect of enhanced miRNA-223 on ox-LDL-induced [Ca^2+^]_i_ generation. [Ca^2+^]_i_ formation was measured with or without ox-LDL treatment for 10, 20, 40, and 60 min. A “dose-response” relationship was observed between Cav1.2 protein and ox-LDL levels. Bars represent mean ± SD of quantitative densitometric analyses from four separate experiments, **P < 0.001 vs. Ctl, *P < 0.01 vs. Ctl, ^†^*P* < 0.05 vs. Ctl. (**E**) Cav1.2 protein expression was measured at 30 min after 25 μg/mL ox-LDL treatment or without ox-LDL treatment. *P < 0.01 vs. Ctl. (**F**) Left, verification of Cav1.2 protein expression changes by western blotting. Right, Cav1.2 expression changes were higher in Tg mice exposed to ox-LDL than in NC mice, *P < 0.001. Ctl, mock-treated with ox-LDL; AMO, antisense oligonucleotides against miR-223; NC, negative control.

**Figure 3:** MiRNA-223 loss-of-function. (**A**) AF induction was substantially dampened in adv-miRNA-223-treated WT mice. (**B**) Surface electrocardiograms (ECG) detected changed spontaneous sustained AF in antagomiR-223-treated AMO/Tg mice. (**C**) Adv-miR-free, adenovirus vector without miRNA-223 (NC construct) knockdown in WT mice. (**D**) The above changes were not observed in WT mice treated with mismatched AMO/Tg mice. (**E**) Levels of miRNA-223 protein and mRNA were increased 2-fold in AF mice (*P < 0.05 vs. WT). (**F**) MiRNA-223 mRNA and protein expression were decreased in miRNA-223 knockdown mice (**P < 0.01).

**Figure 4:** *CACNA1C*/Cav1.2 as the target gene for miR-223. (**A**) Luciferase assays in H9c2 cells for posttranscriptional excitation of *CACNA1C* (the gene encoding cardiac L-type Ca^2+^ channel αlc (Cav1.2) protein). Regulation of Cav1.2 protein expression by miR-223. Western blot showing the effect of miR-223 (*n* = 10) and antisense miR-223 (AMO-223; *n* = 10) on Cav1.2 protein expression in H9c2 rat atrial cells. MiR-223 (10 nmol/L) and AMO-223 (10 nmol/L) were transfected, and then the cells treated with ox-LDL. Ctl, mock-treated with ox-LDL; miR-NC, NC miRNA. **P < 0.001, *P < 0.05 vs. NC; **P > 0.05, *P > 0.05 vs. Ctl; ^+^*P* < 0.05 vs. NC; ^+^*P* < 0.001 vs. Ctl; (**B**) Western blot analysis of Cav1.2 and Cav β1 proteins in atrial tissues from miR-223 Tg and WT mice. **P < 0.001 vs WT, unpaired *t* test; *n* = 10 mice in each group. *P < 0.05 vs. Ctl. (**C**) Western blot analysis of Cav1.2 and Cav β1 proteins in atrial tissues from A-TP dogs. Connexin 43 protein (Cx43) was used as the NC. **P < 0.001 vs. Ctl, unpaired *t* test; *n* = 10 protein samples from two dogs in each group. *P < 0.05 vs. Ctl. (**D**) Effect of miR-223 on Cav1.2 and Cav β1 transcript levels in miR-223/Tg mice and cultured neonatal rat atrial myocytes. *n* = 10 RNA samples in each group. **P < 0.001 vs Ctl, *P < 0.05 vs. Ctl, unpaired *t* test. (**E**) Cav1.2 and Cav β1 protein upregulation in atrial tissues from AF patients with rheumatic heart disease compared with non-AF subjects (Ctl). **P < 0.001 vs Ctl, unpaired *t* test; *n* = 20 patients in each group. *P < 0.05 vs. Ctl.
